The article "Environmental protection in selected one belt one road economies through institutional quality: Prospering transportation and industrialization" was retracted in 2024. Reasons: compromised peer review; unreliable data; unreliable results or conclusions; concerns about the data.

# Environmental protection in selected one belt one road economies through institutional quality: Prospering transportation and industrialization

**DOI:** 10.1371/journal.pone.0240851

**Published:** 2021-01-14

**Authors:** Qiong Wu, Ghulam Rasool Madni

**Affiliations:** 1 International Cooperation Division, Taiyuan University of Technology, Taiyuan, China; 2 Department of Economics and Business Administration, University of Education, Lahore, Pakistan; Institute for Advanced Sustainability Studies, GERMANY

## Abstract

The effects of economic development on natural environment is explored by momentous literature, this study focuses on exploring the role of institutional quality for environmental protection in the selected One Belt One Road (OBOR) economies. The main goal of the paper is to find the threshold level of institutional quality that may minimize CO_2_ emissions in the atmosphere due to widespread industrialization and transportation. The data is selected for the panel of 33 OBOR economies over the time period of 1986–2018. The panel threshold regression technique is applied to determine the threshold level of institutional quality. The estimated results of the study reveal that 2.315 is the threshold level of institutional quality in selected partner OBOR countries. If quality of institutions is above the threshold level then CO_2_ emission do not contribute significantly for environmental deterioration in spite of growing industrialization and transportation and vice versa. The study emphasized to improve the institutional quality up to threshold level to get potential gains from industrialization and transportation.

## Introduction

Environmental deterioration is a burning issue and dreadful problem for the world now days. The global economies are facing serious climatic challenges with economic and social consequences. The greenhouse gases emitting from fossil fuels used for energy, transportation and production purposes; are posing serious effects on natural environment. Long term and durable solutions are required by entire economic agents to reduce these emissions. The transformation of energy, social and economic systems have fundamental role for transition towards low carbon economy. The targeted environmental, social and economic policies have crucial importance for steering such transition but institutional quality is needed to be combined for assurance and implementation of these policies effectively [1]. This study is an attempt to explore the importance of institutional quality in combination with industrialization and transportation for environmental performance in selected OBOR economies.

International trade is growing day by day and there is search for international trade partners. For the purpose, China started the One Belt One Road (OBOR) project in 2013 to create economic and institutional relations through developing the trade networks among Middle East, Asia, Europe and Africa. The estimated cost for this project is $ 21.1 trillion benefitting more than sixty-five countries having the 80% of world population [2–3]. The OBOR project is a source of encouragement for trade and efficient resource allocation as well as maintaining economic growth but environmental deterioration is also a greater threat in the region [4–6].

The article "Environmental protection in selected one belt one road economies through institutional quality: Prospering transportation and industrialization" was retracted in 2024. Reasons: compromised peer review; unreliable data; unreliable results or conclusions; concerns about the data.

Transportation makes possible the distribution of resources across the globe but it is also contributing to environmental deterioration through emissions of CO_2_, Hydrocarbons, Methane, Nitrous Oxide (N_2_O) and discharged water vapors; causing to increase the atmospheric temperature. The actual effects of these gases in the atmosphere of earth are not sure but the “Intergovernmental Panel on Climate Change (IPCC) has predicted that doubling of CO_2_ concentrations could lead to a rise in sea levels by 3.5–5.5 cm per decade due to thermal expansion of ocean waters and melting ice caps and glaciers” [6]. In recent decades, the environmental and social effects of transportation became a topic of interest for researchers and policy makers. The problem of environmental quality and transportation is paradoxical in nature [7]. Since transportation is a source to convey substantial socio-economic benefits while on the other side, it has deep influence to deteriorate the environmental quality. The Fig 1 shows the per capita greenhouse gas emissions in different countries from transportation industry in 2017.

**Fig 1:** Per capita greenhouse gas emissions from transportation industry in 2017. Source: World Development Indicators.

In the literature, it is highlighted that increase in per capita income, freight transport and industrialization have significant role for environmental deterioration and CO_2_ emissions is one of the most challenging task for the society of 21^st^ century [7–9].

The importance of industrialization cannot be negated for economic development and growth but harmful effects for the environmental quality are highlighted in literature massively. Industrial process is causing for environmental change; pollution to soil, water and air; extinction of species; health issues and many more [9]. The global CO_2_ emissions by sectors is given in Fig 2.

**Fig 2:** Global CO_2_ emissions by sectors. Source: World Development Indicators.

Realizing the severity of the issue, impact of industrialization on the environmental quality is needed to be analyzed in further depth. The use of green approaches based on 6R’s technologies (rethink, redesign, recovery, recycle, reuse, reduce) and closed loop systems equipped with industrial ecology provide excellent opportunities to save natural resources. The economic growth of South Asian countries is heavily dependent on industrial sector since last three decades [10]. The manufacturing sector of Thailand and Malaysia contributed 30% in their GDP’s in the decade of 90’s while Indonesia and Philippines have 20% share in their GDP’s in the same period. On the other hand, CO_2_ emissions of developed economies are 70% of world’s carbon dioxide in 1960’s [10–14]. In industrial sector, utilization of fossil fuels is main source of energy; causing to increase the level of CO_2_ emissions tremendously. The industrial sector emits 37% of Green House Gases (GHG); accounts for 80% utilization of energy. The utilization of fossil fuel is reducing the natural reserves of earth on the one side and causing the environmental deterioration, climate change on the other side [15–19].

The article "Environmental protection in selected one belt one road economies through institutional quality: Prospering transportation and industrialization" was retracted in 2024. Reasons: compromised peer review; unreliable data; unreliable results or conclusions; concerns about the data.

Institutions are the informal norms and formal rules of a society and play a significant role for protection of environmental quality while getting the potential benefits from transportation and industrialization [6]. The constructive impact of institutions for sustained functioning of economies cannot be negated now days as supported by massive literature [20–23]. The institutional quality in a country may be a key factor for perseverance of environment. So, institutions should be treated as input for sound legislation and effective implementation to improve the environmental quality across the globe [24]. Institutions are combination of rules, rights and decision making through organizations that emphasize more on environmental quality. The highest level of human security is gained when communities and individuals have aim to decrease threat to human life by promoting environmental quality and social rights. Efficient institutions may affect growth and environmental quality by guaranteeing the environment friendly industries. High quality institutions provide the freedom to people for their political and information rights. This freedom establishes the groups and organizations having environmental interests and source for public awareness regarding preserving the natural environment which encourage the environmental legislation. On the other hand, inefficient institutions fail to implement environmental friendly approaches in the society. The environmental protection cannot be assured without political authorities [8, 12, 24]. It can be hypothesized that a certain level of institutional quality is helpful to reduce the level of CO_2_ emission and hence reducing the environmental deterioration. The threshold level of institutional quality to overcome the environmental challenges is hardly explored in the literature; the prime objective of the study.

The article "Environmental protection in selected one belt one road economies through institutional quality: Prospering transportation and industrialization" was retracted in 2024. Reasons: compromised peer review; unreliable data; unreliable results or conclusions; concerns about the data.

The motivation to examine the relationship among CO_2_ emission, institutions, transportation and industrialization is that; OBOR project will not only increase the income of partner economies but reduced trade cost will also increase the real income of other countries of the world. According to Belt and Road Portal [25], the global real income will be increased by 0.7% till 2030 through one belt one road and host countries will get the benefit of 70% of this raise. In addition, this project will increase the economic growth of partner countries also as the partner countries of OBOR hold the half of global GDP but on the other side, the CO_2_ emission of these countries accounts for 54% of global Carbon Dioxide emissions. It is recorded that major portion of energy generation in OBOR partner countries is carried through coal based projects and these countries spend 65% of their energy generation budget on coal based projects. Only China is responsible for spending of 40% public investment in coal based projects globally from 2007 to 2014. The 240 coal based energy generation plants are installed in 25 OBOR partner countries having capacity to produce 251 Giga watts energy and many firms of China are intended to install more 92 coal based plants in 27 partner economies of OBOR project. It will increase the emission of Carbon Dioxide by further 62% in partner countries of OBOR project as described by BP Statistical Review of World Energy 2017. A comparative pattern of CO_2_ emissions in OBOR economies and whole world is shown in Fig 3.

**Fig 3:** CO_2_ emission in belt and road initiative economies and world. Source: World Development Indicators.

In 2014, China, India and Russian were emitting CO_2_ in global atmosphere with contribution of 28%, 6% and 5% respectively while the OBOR project will further increase the Carbon Dioxide in the air. In 2014, GDP of collaborating countries is 45% of global GDP while energy consumption is equivalent to half of global energy consumption and CO_2_ emissions are 54% of the globe. The OBOR project is also considered as to deteriorate environmental quality in future [26–28]. It can be concluded that partner countries of OBOR project will excel their economic growth in future resultantly leading to pollute environment further. It is dire need of time to investigate the strategies helpful to slow down the environmental degradation without compromising the living standard of people. It is also a great challenge and important to know for collaborating countries to develop a strategy for reduction of CO_2_ while getting the potential benefits of OBOR project with special reference to growing industrialization and transportation. Global shifting wave for OBOR projects will pose adverse impact on natural resources and ecosystem [29–30]. Institutional quality in partner countries may play a significant role for environmental protection. However, relation among transportation, industrialization and environmental quality has been investigated for partner countries of OBOR project in literature but role of institutional quality is still largely absent. This study is an attempt to determine the threshold level of institutional quality that may be helpful to minimize the CO_2_ emission. The threshold effect allows the asymmetric effect of independent variables depending on whether the threshold variable is below or above the unknown threshold. This study is an attempt to provide empirical evidence about the threshold level of institutions that may influence the quality of environment in selected OBOR countries. It is examined that how relationship between CO_2_ emission and other variables vary along with changes in institutional quality. Specifically, the study has objective to determine the threshold level of institutions which may bring the fruits of industrialization and transportation along with environment protection. To our best knowledge, there is hardly any study exploring the threshold level of institutional quality to control the adverse effects on environment for OBOR partner countries; the central objective of this paper. The extent of this relationship varies with changes in institutional quality. Finding the threshold level of institutional quality may have beneficial policy implications for reduction of CO_2_ emissions as well as economic expansion through industrialization and transportation.

The article "Environmental protection in selected one belt one road economies through institutional quality: Prospering transportation and industrialization" was retracted in 2024. Reasons: compromised peer review; unreliable data; unreliable results or conclusions; concerns about the data.

## Literature review

The earlier below studies highlight the effects of industrialization and transportation for environmental deterioration but role of institutions is highlighted very little. The institutional quality up to a certain level will be helpful for environmental protection in spite of industrialization and rapidly expanding transportation. The relationship between environmental quality and growth initially is elaborated [31]; later on it was termed as “Environmental Kuznets Curve” (EKC). EKC discusses that increase in growth deteriorates environmental quality at earlier stages but then it will upgrade the environmental quality with increase in economic growth. Policy makers design the environment friendly policies that further decrease the green house gases and CO_2_ emission. These policies include consumption of renewable energy, inducement of mechanism which is energy efficient, induction of treatment plants in industry. Environmental Kuznets Curve shows the inverted U shaped curve showing relation between environmental quality and growth. Many studies [11, 32–37] empirically proved presence of Environmental Kuznets Curve in many countries.

According to [38], major Taiwan industry is emitting carbon dioxide extensively deteriorating environmental quality while [39] found that industrialization in developed countries is causing for degradation of environment. The industrial, agricultural and services sectors of Turkish economy for the period of 1970–2006 are investigated [40] to determine the factor that may cause to alter the level of CO_2_ emissions. The findings of the paper pointed out that CO_2_ emission kept on rising because of rapid expansion of industry so industrialization is a main source to raise the level of carbon dioxide emissions. The study [37] highlighted that expansion of industry deteriorates the environment at earlier stage of development then after at certain level, industrial expansion will not deteriorate environmental quality in Bangladesh.

Transport sector is a major source deteriorating the quality of environment but travelling behavior affect CO_2_ emissions [41]. The findings of [42–45] elucidate that many people live in territory having greater opportunities of employment and this employment creates residential density. These dense areas emit CO2 in atmosphere extensively. The availability and usage of public transport enhances the environmental quality. It can be concluded that travelling behavior and provision of public transit service have greater importance for environment [46–50].

The study [51] explored the relationship among institutions, economic growth and CO_2_ emission in Malaysia by considering the sample period of 1984–2008 and applied bounds testing technique. The findings of the study reveal that institutions, CO_2_ emissions positively affect the economic growth. It is further investigated that institutional quality may play its role for reduction of CO_2_ emission in Malaysia. This improvement in environmental quality would increase the level of economic development. It is concluded that institutional structure affects the level of economic growth both indirectly and directly along with reduction of CO_2_ emission. The findings of other studies also reveal that institutional quality enhance environmental quality [24, 52].

The study [53] used panel co-integration technique to examine the relationship among climate change, air pollution, and energy consumption for panel of 6 economically diversified countries. The empirical findings of the study highlighted that “energy consumption and air quality have positive and substantial impact on climate change. The results further highlight that 1% increase in energy consumption raises the emission of greenhouse gases by 0.124%, carbon dioxide emissions by 0.652%, methane emissions by 0.123%, and nitrous oxide emissions enhances greenhouse gas emissions by 0.105%. However, the fixed and random effect regression result proved the weakening of air quality indicators on climate change.”

The article "Environmental protection in selected one belt one road economies through institutional quality: Prospering transportation and industrialization" was retracted in 2024. Reasons: compromised peer review; unreliable data; unreliable results or conclusions; concerns about the data.

The effect of Environmental Kuznets Curve for CO_2_ emissions in eleven countries is investigated for the period of 1990–2014 by segregating the forms of energy into non renewable, renewable and biomass energy [54]. The Generalized Method of Moments (GMM) is applied for empirical investigation and found the N-shaped relation for environmental deterioration and growth for sample countries. The interactional impact among economic growth, biomass energy and trade openness is further analyzed and found negative relationship for CO_2_ emission.

The impact of urbanization on environment is investigated for Singapore because all population of Singapore is urban [55]. The study shows negative relationship of urbanization with CO_2_ emission which conveys that urbanization does not matter for environmental deterioration. On the other hand, economic growth plays its role for environmental degradation. The main empirical findings show that renewable energy increase the growth but do not contribute to deteriorate the environment [56]. The study applied robust panel econometric technique for period of 1990–2012 to examine the relationship among renewable energy consumption, economic growth and CO_2_ emissions of the fastest developing economies.

The relationship among economic growth, transportation infrastructures, trade, labor, education and inflation in One Belt One Road Initiative countries is investigated [57]. The study used the annual panel data for the period of 2000 to 2015 for the selected Asian countries by dividing into three regions. The results through fixed effect model divulge that transportation infrastructure affects the economic growth positively in these countries while education is not contributing significantly for GDP. It is suggested for policy makers to upgrade their system in context of education, human capital and transportation infrastructure in OBOR partner countries.

The study [58] highlighted the “relationship between industrial value added per capita, transport freight and CO_2_ emission among the partner countries of Belt and Road initiatives by using panel of 33 economies from 1986–2017. Estimated results of pool mean group (PMG) indicate that increase in industrialization and transportation deteriorates the quality of environment in long run. However, short run results of granger causality reveal positive and unidirectional causality running from industrial value added per capita to emission of CO_2_ while transport freight and CO_2_ emission shows bidirectional causality. The study emphasized to formulate environment friendly policies in industrial and transport sector.”

The article "Environmental protection in selected one belt one road economies through institutional quality: Prospering transportation and industrialization" was retracted in 2024. Reasons: compromised peer review; unreliable data; unreliable results or conclusions; concerns about the data.

The study [59] explored the impact of infrastructural development on environmental quality as well as on social, political and economic factors in China’s Belt and Road Initiative economies. In this study, authors also developed a typology for Belt and Road Initiative infrastructure explaining the effects of different components of atmosphere and other socio-economic and political factors that influence the Belt and Road Initiative projects. The study argued that a multi scale approach is required for analysis of environmental impact by the Belt and Road Initiative and to devise a policy and plan for addressing its impacts. A single approach is not helpful which may embody the cumulative impacts of this project on environment.

## Data description and methodology

The study selected the annual data for sample of 33 OBOR countries for time span of 1986–2017. This sample is adopted due to availability of data from International Country Risk Guide (ICRG) and World Development Indicators (WDI). The model of the study is extension of [60] to explore the relationship among CO_2_ emission, institutional quality, industrialization, transportation and control variables.

$$CO_{2}=f\left(Institutions,\;Industrialization,\;Agriculture,\;GDP,\;Trade,\;Transportation\right)$$

Institutions have their significance for economic performance of any country. The efficient and strong institutions assure the effective implementation of environmental policies by government. If institutional quality is low in any country, then profit seeker firms pay briberies to officials for using of machinery and technology that pollute the environment [48]. Because environmental polluting plants are cheaper as compared with environmental friendly plants and technology so firms prefer them to maximize their profits. It can be hypothesized that inefficient institutions are barrier in the way of cleaner atmosphere [22, 47–49]. In developing countries, low per capita income puts pressure on political governments to enhance their economic growth instead of focusing on environmental issues. The inefficient institutions in developing economies sacrifice environmental quality for the sake of economic development [57]. The low quality institutions remain less efficient to control CO_2_ emission as compared with developed economies [45]. It can be argued that improvement of institutional quality may be a source to increase economic growth and higher income level increase the awareness about green challenges and control of green house gases. In addition, implementation of competition in emerging economies increases the efficiency leading to decrease the level of CO_2_ emissions [55]. However, emerging economies focus more and more on environmental challenges as the per capita income increases [42]. The high quality institutions attract foreign direct investment in the country so there is rapid expansion in trade, transportation, industrialization and hence economic growth. It is important to determine the level of institutional quality which is helpful to boost these economic activities without compromising on the green environment. If institutions are not up to a certain level, then economic expansion will lead to deteriorate the quality of environment. This study is an attempt to determine threshold level of institutional quality in selected OBOR partner countries which will be a source of economic expansion with lower level of environmental degradation.

The article "Environmental protection in selected one belt one road economies through institutional quality: Prospering transportation and industrialization" was retracted in 2024. Reasons: compromised peer review; unreliable data; unreliable results or conclusions; concerns about the data.

It is evident that industrialization, economic growth, trade and transportation are the sources to pollute the environment [13]. These economic activities emit numerous toxic gases like Carbon Dioxide, Methane, Carbon Monoxide, Nitrous Oxide, Chlorofluorocarbons and polluting the environment in several aspects [58]. Vehicles are also big contributor of pollution in atmosphere along with occupying the 23–29% of agricultural land and natural habitats [61]. Moreover, agriculture sector is harming the environment less as compared with other sectors of the economy like transport and industry [58].

The natural logarithm is applied for linear specification because linear specification provides reliable and efficient estimation as compared with other specifications [62–64]. Furthermore, CO_2_ emission is proxy for environmental quality measured as per capita metric tons, industrialization and agriculture are value added as percentage of GDP, GDP is per capita GDP, trade is percentage of GDP and transportation is movement of goods through inland transport measured in millions tons per kilometer. The variable of institutional quality is constructed through Principal Component Analysis (PCA) for twelve clusters of indicators of institutions from International Country Risk Guide (ICRG). These indicators have range from 0 to 10 means higher score reflects higher condition and vice versa. The details of variables are given in Table *1*.

The article "Environmental protection in selected one belt one road economies through institutional quality: Prospering transportation and industrialization" was retracted in 2024. Reasons: compromised peer review; unreliable data; unreliable results or conclusions; concerns about the data.

**Table 1:** Description of variables.

Variables	Measured	Source
CO_2_ Emission	Per Capita Metric Ton	WDI
Institutions	Index of Twelve Indicators	ICRG
Industrialization	Value Added as % of GDP	WDI
Agriculture	Value Added as % of GDP	WDI
GDP	Per Capita GDP	WDI
Trade	As Percentage of GDP	WDI
Transportation	Movement of goods through inland transport measured in millions tons/kilometer	WDI

The empirical equation can be written as follows.

$$CO_{2it}=\beta_{0}+\beta_{1}\;INSQ_{it}+\beta_{2}\;INDS_{it}+\beta_{3}\;AGRI_{it}+\beta_{4}\;GDPP_{it}+\beta_{5}\;TRAD_{it}+\beta_{6}TRNS_{it}{}_{}+\varepsilon_{it}$$ (1)

Based on the threshold regression technique, Eq (2) is derived to capture the affect of industrialization and transportation on CO_2_ emissions in presence of contingency effects.

$$CO_{2it}=\left\{ \begin{array}{c} \beta_{0}^{1}+\beta_{1}^{1}INDSit+\beta_{1}^{1}TRNSit+\beta_{3}^{1}Xit+eit,\;INSQ\leq \phi \\ \beta_{0}^{1}+\beta_{1}^{2}INDSit+\beta_{1}^{2}TRNSit+\beta_{2}^{2}Xit+eit,\;INSQ>\phi \end{array}\right.$$ (2)

In above equation, INSQ is the threshold variable representing institutional quality and utilized to split the sample into groups or regimes while vector of control variables is shown by *X* and ϕ is symbolized for unidentified threshold parameter. $\beta_{1}^{1}$ is for low regime countries and $\beta_{1}^{2}$ is for higher regime countries. According to hypothesis of the study, β^1^ = β^2^ so prescribed model is again linear and demotes to Eq (1).

Null hypothesis of linearity *H*_*0*_: *β*_*1*_ *= β*_*2*_ is tested for Eq (2) in first step of estimation. The non standard inference problem emerges due to non identification of threshold parameter under the null hypothesis so Lagrange Multiplier or Wald test do not hold conventional chi-square limits as pointed out [65–66]. Instead, super mum of the LM or Wald test statistics is calculated to implement the inferences for all possible values of ϕ. This limiting distribution of nonstandard super mum statistics depends upon many nuisance parameters so inferences are implemented through a bootstrap model established [65]. The study [66] suggested a technique of instrumental variable threshold regression to deal with problems of endogeneity and threshold non linearity so Eq (1) takes the following form;

$$CO_{2it}=\left(\beta_{1}\;INDS_{it}+\beta_{1}TRNS_{it}+\alpha_{1}X_{it}\right)1(INSQ_{it}\leq \phi )+\left(\beta_{2}INDS_{it}+\beta_{2}TRNS_{it}+\alpha_{2}X_{it}\right)1(INTQ>\phi )+\varepsilon_{i}$$ (3)

$$INDS_{it}=\left(\gamma_{1}\;Z_{it}+\mu_{1}\;X_{it}\right)\;1\;\left(INSQ_{it}\leq \phi \right)+\left(\gamma_{2}\;Y_{it}+\mu_{2}\;X_{it}\right)\;1\;(INSQ>\phi )+v_{i}$$ (4)

Where 1(·) and *Y* represent indicator function and a vector of instrumental variables respectively, satisfying the order condition. To estimate the regression coefficients, a three step procedure is suggested [66]. In first step, ordinary least square method is applied to get the fitted values of *INDS*_*i*_ and *TRNS*_*i*_ by regressing it on instrumental variables. Government expenditure is considered as an instrumental variable as cross country differences linking the CO_2_ emissions and industrialization. The next step is substitution of predicted values of *INDS*_*i*_ and *TRNS*_*i*_ into Eq (3). The third step is again applying of ordinary least square method to estimate the threshold parameter ϕ. Finally, on basis of threshold parameter, the whole sample is divided into two sub samples and generalized method of moments is applied to obtain the slope parameters. Then super mum Wald statistics is tested for existence of threshold level and derived the asymptotic distribution.

The article "Environmental protection in selected one belt one road economies through institutional quality: Prospering transportation and industrialization" was retracted in 2024. Reasons: compromised peer review; unreliable data; unreliable results or conclusions; concerns about the data.

## Empirical findings

Table 2 describes the descriptive statistics comprising on mean, standard deviation, maximum and minimum values of variables.

**Table 2:** Descriptive statistics.

Variable	Unit	Mean	Std. Deviation	Max	Min
CO_2_	Per Capita Metric Ton	5.74	4.54	18.25	0.33
GDP	Per Capita GDP	10716.6	12801	60913.7	806.4
Industrialization	Value Added as % of GDP	30.25	10.20	59.72	9.27
Agriculture	Value Added as % of GDP	8.78	7.53	30.07	0.09
Trade	As Percentage of GDP	80.65	59.73	329.4	21.33
Institutions	Index of Twelve Indicators	4.94	2.39	9.98	2.01
Transportation	Movement of goods through inland transport measured in millions tons/kilometer	7.28	4.51	21.38	0.85

After finding the descriptive statistics of the variables, Eq (2) is estimated and results are shown in Table 3. Bootstrap method is used to evaluate the p-value for significance of threshold estimate.

**Table 3:** Threshold estimates of institutional quality.

	Ethnic Diversity
**First Sample Split**	
Threshold Estimate	2.315
Bootstrap p-value	0.002
LM test for no threshold	19.71
95% Confidence Interval	(2.619, 2.837)
**Second Sample Split**	
Bootstrap p-value	0.759
LM test for no threshold	5.33

Note: Null hypothesis: No threshold effect.

The p-values of model indicate that null hypothesis of no threshold effect cannot be accepted so presence of threshold effect can be found for such analysis. On the basis of estimated results, sample can be divided into two regimes or groups. The threshold value of institution is 2.315 with 95% confidence interval of (2.619, 2.837). It can be concluded that countries having institutional quality below than 2.315 are classified as low institutional quality group while countries above this value are considered as high institutional quality group.

The article "Environmental protection in selected one belt one road economies through institutional quality: Prospering transportation and industrialization" was retracted in 2024. Reasons: compromised peer review; unreliable data; unreliable results or conclusions; concerns about the data.

After finding the presence of threshold effect for institutional quality in the model, how institutions affect the relationship between CO_2_ emissions and industrialization is a question to be answered. For this purpose, a model for indicator of industrialization is regressed and estimated results are reported in the Table 4. In this model, institutional quality is a threshold variable while CO_2_ emissions is a dependent variable. The Table 5 presents the empirical findings gained through instrumental variable threshold regression technique.

**Table 4:** Results using OLS threshold regression.

	Linear Model	Threshold Model	
	OLS	Group 1	Group 2
		INSQ ≥ 2.527	INSQ ≤ 2.527
Constant	2.916** (0.371)	1.927* (0.249)	3.862* (1.729)
INDS	0.36 (0.144)	0.648** (0.194)	0.073 (0.157)
AGRI	-0.191** (0.121)	-0.433** (0.391)	-0.725* (0.644)
GDPP	1.151** (0.199)	1.726** (0.661)	2. 114 (0.394)
TRAD	0.261 (0.073)	0.262 (0.138)	0.317 (0.261)
TRNS	0.249 (1.481)	0.228*** (1.174)	0.192 (1.384)
INSQ	-0.381** (0.243)	-0.418 (0.463)	-0.861** (0.253)
R^2^	0.74	0.48	0.68

Note

*, **, *** show significance at 1%, 5% and 10% respectively.

**Table 5:** Results of instrumental variable threshold regression.

	Threshold Model	
	Group 1	Group 2
	INTQ ≥ 2.642	INTQ ≤ 2.642
Constant	1.427* (0.374)	4.482* (1.896)
INDS	0.234* (0.172)	0.193 (0.241)
AGRI	-0.270* (0.136)	-0. 831* (0.381)
GDPP	2.417* (0.317)	1.317* (0.471)
TRAD	0.168 (0.134)	0.762 (0.537)
TRNS	0.184** (1.433)	0.083 (2.473)
INSQ	-0.382 (0.251)	-0.793* (0.442)
R^2^	0.45	0.59

Note

*, ** show significance at 1% and 5% respectively.

Tables 4 and 5 present the empirical findings showing the relationship among institutional quality, CO2 emissions, industrialization and transportation. To deal with problems of endogeneity and threshold non linearity, instrumental variable threshold regression technique is applied proposed by [66] and findings are reported in Table 5. Government expenditures are used as an instrumental variable. The value of super Wald test statistics is 66.492 (0.000) significant at 5% showing the significant presence of a threshold effect in relationship of CO2 emissions, industrialization and transportation; suggesting two separate groups of countries with respect to their prevailing institutional quality. It can be found from empirical results that in group with high quality institutions; industrialization and transportation do not contribute significantly to pollute the environment. If institutional quality falls below the threshold level in the countries then industrialization, per capita GDP and transportation are playing their significant role to deteriorate the environmental quality. On the other side, institutional quality and agriculture sector have positive relationship in the OBOR economies.

The article "Environmental protection in selected one belt one road economies through institutional quality: Prospering transportation and industrialization" was retracted in 2024. Reasons: compromised peer review; unreliable data; unreliable results or conclusions; concerns about the data.

The reported results point out that industrialization, transportation and per capita GDP contribute significantly to increase the CO_2_ emission if institutional quality is below the threshold level and if the countries having the institutional quality above the threshold level then industrialization, transportation and per capita GDP do not contribute significantly to increase emission of carbon dioxide. The empirical findings highlight that institutional quality in the OBOR countries has crucial importance for environmental protection. The institutional quality above the threshold level may contribute to improve the living standard of people through industrialization and transportation while environmental degradations remain unaffected while below the threshold level of institutional quality; any effort to enhance the industrialization would cause to deteriorate the environmental quality due to emissions of carbon dioxide. It can be argued that better quality institutions are a barrier in the way of environmental deterioration. The high quality institutions attract foreign direct investment in the country so there is rapid expansion in transportation, industrialization and hence economic growth. These economic activities pollute the environment if institutional quality lies below the threshold level while environment is less polluted if institutional quality is above the threshold level. It can be explained in many ways; the emerging economies prefer improvement of economic institutions that boost their economic growth while institutions dealing with environmental performance remain at their least priority [33, 52, 58]. The inverse relationship between environmental protection and economic growth is a greater challenge for leaders of developing countries. There is dire need to improve the quality of economic institutions as well as environmental protection institutions at the same time. It will attract FDI on the one side and this FDI will be a source to develop environment friendly technology leading to less polluted environment [26]. With the advent of FDI in a country due to high quality institutions, the per capita income of people will rise as well as their awareness for green environment demanding environmental friendly policies regarding industrialization and transportation. Mere improvement of economic institutions will increase emission of CO_2_ in atmosphere. It is suggested for policy makers to undertake institutional reforms and bring the quality of institutions up to threshold level for a less pollutant environment. The low quality institutions are suppressing their economic growth and polluting the global environment [55]. All above can be concluded that institutional quality up to threshold level is necessary for environmental protection then expansion of industrialization and transportation may have less harmful effects to environment.

The article "Environmental protection in selected one belt one road economies through institutional quality: Prospering transportation and industrialization" was retracted in 2024. Reasons: compromised peer review; unreliable data; unreliable results or conclusions; concerns about the data.

The transportation is considered as the most important birthplace of CO_2_ emission due to combustion of fossil fuels. Rapidly increasing services of transport sector are causing many environmental and societal issues. The transport share for CO_2_ emission increased from 21% to 23% in the period of 1991–2007 and its share will increase to 23.2% by 2030 approximately. Moreover, demand for transportation is rapidly increasing with expansion of economic activities, which is further increasing the CO_2_ emission and causing to deteriorate the environmental quality. Institutional quality may play its significant role to reduce the harmful effects of widely expanding transportation across the globe.

There is negative relationship between carbon dioxide emissions and agriculture sector in selected OBOR partner countries. Institutions matter for environmental performance but usage of modern farming methods and organic seeds in agriculture sector are helpful to decrease the level of CO_2_ emissions in the atmosphere. According to findings of [58], many countries like Kazakhstan, Russia, Tajikistan and Uzbekistan are intended to reduce the quantity of pesticides and nitrogen rich fertilizer in agriculture sector by 10 percent. Moreover, utilization of natural water may have impact to decrease the greenhouse gas emissions in the region. The latest farming techniques are also a source to slow down the rate of soil erosion [45, 58]. It is elucidated that agriculture sector is less polluting sector as compared with other sectors of the economy.

Industrialization is an important engine of economic growth in any country but it is also polluting the environment as empirical findings are reported. It is estimated that 30% of global greenhouse gases comes from industry [57]. OBOR partner countries have many outdated technologies and environmental polluting infrastructure for industry [48]. The industrialization process expands until saturation of industrial development then it declines [56]. The declining trend of industrial expansion brings the modern environmental friendly technologies but it depends upon the prevailing institutional quality in the country. If institutional quality is higher then industrialization process promotes green industry and vice versa. The environmental regulations or ordinances and their effective implementation bound the firms for utilization of green technologies, hence environmental deterioration slows down.

The article "Environmental protection in selected one belt one road economies through institutional quality: Prospering transportation and industrialization" was retracted in 2024. Reasons: compromised peer review; unreliable data; unreliable results or conclusions; concerns about the data.

All above discussion conveys that the institutional quality matters a great for environmental protection in the OBOR countries. If we have a look upon the findings of earlier studies then we come to know that the OBOR project will deteriorate environmental quality in host countries [29–30, 67–69]. The growing industrialization is a source of environmental degradation due to extensive emission of by-products, smoke and materials. The by-products include the toxic elements which are dangerous for human lives as well as for earth. If institutional quality in these countries lies at above the threshold level, then industrialization and transportation will not deteriorate the environmental quality significantly. These findings are also in line with findings of [45, 51, 52, 58] who found that institutional quality play significant role to reduce CO_2_ emissions.

## Conclusions and policy implications

Environmental protection requires a fundamental change in economic as well as social policies. One Belt One Road project is initiated by China to develop the relations among host economies in sectors of trade and energy. Besides uncountable benefits, transportation and industrialization have a considerable role on environment. This study explores the relationship between institutional quality and other variables concerned to environmental performance. The threshold level of institutional quality for environmental protection is determined. This threshold level of institutional quality slows down the process of environmental deterioration even in presence of ever growing industrialization and transportation in the 33 partner economies of one belt one road project over the time period of 1986–2018. The panel threshold regression technique is applied to determine the threshold level of institutional quality. The findings of the study elucidate that 2.315 is threshold level of institutional quality in sample countries so countries having institutional quality below than 2.315 are classified as low institutional quality group while countries above this value are considered as high institutional quality group. The estimated empirical results highlight that industrialization, transportation and per capita GDP contribute significantly to increase the CO_2_ emission if institutional quality is below the threshold level while industrialization, transportation and per capita GDP do not contribute significantly to increase the CO2 emission in the countries where the institutional quality is above the threshold level. The policy implications based on empirical findings are that, developing economies are required to improve institutional quality in their countries to decrease environmental deterioration due to greenhouse gases. It is necessary to strengthen and improvement of institutional quality and let them function efficiently to preserve the natural environment. Efficient institutions in economies will deliver effective regulations, laws, property rights which will lead to reduce CO_2_ emissions. Moreover, governments in these countries may focus on proper legislation to encourage the consumption of green energy that has minor environmental problems.

The article "Environmental protection in selected one belt one road economies through institutional quality: Prospering transportation and industrialization" was retracted in 2024. Reasons: compromised peer review; unreliable data; unreliable results or conclusions; concerns about the data.

However, there are some limitations of this study. Firstly, the variable of the institutional quality may be strengthened by incorporating more indicators so that it will draw a more realistic picture for relationship between environment and institutional quality. The second constraint or it may be considered as a proposal for future investigation is to measure the behavior of CO_2_ emissions before and after institutional reforms in the OBOR countries.

## Supporting information

S1 Appendix List of countries. (DOCX)
